The article "Image Segmentation-Based Cervical Spine MRI Images to Evaluate the Treatment of Patients with Chronic Pain" was published in 2022. Journal: Comput Math Methods Med.

# Image Segmentation-Based Cervical Spine MRI Images to Evaluate the Treatment of Patients with Chronic Pain

**DOI:** 10.1155/2022/2648659

**Published:** 2022-06-28

**Authors:** Qingqing Guo, Rongchun Li, Waiping Zhou, Xia Li

**Affiliations:** ^1^Department of Pain Management, Wuhan Fourth Hospital, Puai Hospital, Tongji Medical College, Huazhong University of Science and Technology, Wuhan City 430000, China; ^2^Department of Radiology, Wuhan Fourth Hospital, Puai Hospital, Tongji Medical College, Huazhong University of Science and Technology, Wuhan City 430000, China

## Abstract

The objective of this research was to investigate the application effect of cervical spine magnetic resonance imaging (MRI) image segmentation algorithm guidance in the treatment of chronic pain with cervical epidural puncture. A total of 72 patients with chronic pain were selected and divided into a cervical spine MRI image-guided group (group A) and a blind puncture group with traditional experience (group B). The results showed that the puncture time of group A was 9.9 ± 8.2 (min), while that of group B was 15.2 ± 8.9 (min), so the puncture time of patients in group A was significantly shorter than that of group B (*P* < 0.05). The incidences of pain at the puncture site of patients in group A and group B were 6% and 10%, respectively. The incidence of pain at the puncture site in group A was significantly lower than that in group B (*P* < 0.05). The success rate of the first puncture in group A was 78%, and that in group B was 54%. The success rate of the first puncture in group A was significantly higher than that in group B (*P* < 0.05). The complication rate of group A was 22.22%, and that of group B was 80.56%. The incidence of complications in group A was significantly lower than that in group B (*P* < 0.05). In addition, there was no significant difference in the puncture depth between the two groups (*P* > 0.05). In summary, the guidance of cervical spine MRI image segmentation algorithm can reduce the time and times of puncture and improve the success rate of puncture, thereby reducing the incidence of postoperative complications.

## 1. Introduction

Chronic pain is one of the prevalent health problems in modern society, and thousands of people suffer from back pain, cervical pain, headache, and arthritis [1]. Chronic pain is a relatively common clinical condition with a high incidence, with approximately 15~20% of outpatients suffering from chronic pain. Chronic pain, which usually persists or recurs for more than 3~6 months, has a large impact on people's quality of life and physical and mental health [2, 3]. Cervical epidural catheterization is a common pain treatment method widely used in the diagnosis and treatment of various parts of the human body [4, 5]. With the rapid development of medical imaging diagnosis technology, the emerging and application of C-arm and contrast agent have made a qualitative leap in the accuracy of cervical epidural puncture technique. However, the anatomical structure of the cervical spine is more precise and complex by comparing with the thorax or lumbar segments, so there are still some difficulties and challenges of the cervical epidural puncture technique for the physicians from pain department. Therefore, it is of great significance for clinical treatment and prognosis of patients with chronic diseases to take effective measures to promote the targeting of cervical epidural catheterization and minimize the times of punctures and injuries for patients during the treatment.

MRI image measurement is a key link in image-guided cervical epidural puncture [6]. The image measurement technology based on image storage and transmission is extensively applied in medical image system. The picture archiving and communication systems (PASC) is an integral part of the medical information system, which can obtain medical images for imaging diagnosis. In addition, it also can measure, reconstruct, and calculate the images through the image processing tool of workstation, which can provide effective guidance in clinical treatment practice [7, 8]. In recent years, medical image processing technology has become more and more critical with the rapid development of modern medical image technology. In particular, accurate segmentation of medical images is a crucial step in image processing. Image segmentation is vital for diagnosis, 3-dimensional visualization, and image-guided surgery. The realization of accurate segmentation helps doctors understand the actual condition of patients and make reasonable treatment plans [9]. The gradient vector flow- (GVF-) Snake algorithm has been extensively used as an effective method for medical image segmentation but is sensitive to noise and false edges, so as to limit its application scope [10]. The segmentation method based on knowledge is developed from artificial intelligence technology, and segmentation guided by prior knowledge can realize the limitation of segmentation, thus promoting the stability and accuracy of segmentation [11].

The innovation of this work was to propose a cervical spine MRI image segmentation algorithm, apply it to MRI image segmentation processing to obtain images with high segmentation accuracy, under the guidance of which the cervical epidural puncture and catheterization were performed to treat the chronic pain. The objective of this work was to investigate the application effect of cervical spine MRI image segmentation algorithm guidance in the treatment of chronic pain with cervical epidural puncture. The significance of this work was to provide theoretical basis and reference for the clinical diagnosis and treatment of chronic pain patients.

## 2. Materials and Methods

### 2.1. Research Objects and Their Grouping

A total of 72 patients with chronic pain, admitted to hospital from October 2018 to May 2020, were selected as the research subjects. The male to female ratio was 42 : 30, and the patients ranged in age from 35 to 60 years old. Among them, 20 were postherpetic neuralgia, 28 were cervicogenic headache, and 24 were cervical spondylosis. All patients were divided into a cervical spine MRI image-guided group (group A) and a noncervical spine MRI image-guided group (group B) according to different treatment methods, with 36 cases in each group, and all of which were treated with cervical epidural puncture. This research had been approved by ethics committee of hospital, and the patients and their families signed the informed consent forms.

Inclusion criteria are as follows: (I) patients with complete medical records, (II) patients with ability of smooth communication, and (III) patients who and their families signed the informed consent.

Exclusion criteria are as follows: (I) patients with mental and psychological diseases, (II) patients with tumors, (III) patients with abnormal coagulation function, and (IV) patients with infection.

### 2.2. MRI Examination

1.5T MRI scanner was used for the examination. During the examination, the patient remained in the supine position and wore a special nonmagnetic earphone. The scanning process was as follows. The conventional three-plane positioning was adopted. For the image scanning range, sagittal images should cover the foramen magnum to the T1 plane and the neural foramen on both sides, and cross-sectional images should cover the second cervical vertebral body (C2 vertebral body) to the T1 vertebral body level. For the image scanning parameters, slice thickness was ≤3.0 mm, slice spacing was ≤1.0 cm, and the longest inspection time for required sequence acquisition was ≤35 min.

### 2.3. Therapeutic Methods

The patients of group B were treated by the same experienced physician from pain department according to the previous experience. The 2 cm position near the midpoint of the spinous process space was operated with local infiltration. The puncture needle was inclined to a 75° angle with the skin, and the needle was inserted along the vertebral plate space to enter the epidural space after passing through the yellow ligament.

Before the surgery, the patients of group A underwent cervical spine MRI and anterior and lateral X-ray examination to determine the catheter end position, and the middle part of the pain segment was taken as the catheter end position for this treatment. Then, the best way to enter the epidural space was analyzed, namely, which vertebral plate was the most suitable for entry. Next, the insertion point of skin was selected and determined. In general, the skin insertion point was selected to be the inferior spinous process space of the vertebral plate space of the epidural space. Moreover, the angle was measured between the puncture needle and the patient's trunk plane. Besides, the angle should be determined between the puncture needle and longitudinal section of the body, so as to plan and determine the puncture path. Then, there were determinations of the puncture angle, the length of epidural catheter placement, and the depth of the needle insertion. Finally, the patients received the epidural puncture based on the parameters determined by the above operations.

### 2.4. Cervical Spine Magnetic Resonance Imaging-Based Image Segmentation Algorithm

In this work, the deformable model GVF-Snake was used to segment the vertebrae of the patient's magnetic resonance images. Snake was a curve *L*(*s*) defined within the image area and can be represented as follows.

(1) $$\begin{array}{c} L\left(s\right)=\left(x\left(s\right),y\left(s\right)\right),s\in \left[0,1\right]. \end{array}$$

In equation (1), *x* (*s*) and *y* (*s*) stood for the coordinate positions of the control point.

Snake converged towards the boundary or target mainly by the combined action of internal and external forces. Minimum energy was at equilibrium position. Snake energy function was shown as follows.

(2) $$\begin{array}{c} E=\int_{0}^{1}\frac{1}{2}\left[\alpha {\left|L^{\prime }\left(s\right)\right|}^{2}+\beta {\left|L^{\prime \prime }\left(s\right)\right|}^{2}\right]+E_{\mathrm{ext}}\left(L\left(\text{s}\right)\right)ds=\int_{0}^{1}E_{\mathrm{int}}+E_{\mathrm{ext}}\left(L\left(s\right)\right)ds. \end{array}$$

In equation (2), *E*_ext_ represented the external energy; *E*_int_ expressed the internal energy; |*L*′(*s*)|^2^ and |*L*′′(*s*)|^2^ controlled the Snake elasticity and rigidity in sequence; both *α* and *β* stood for coefficients.

*A*(*x*, *y*) of grayscale image could be expressed as follows.

(3) $$\begin{array}{c} E_{\text{line}}=A\left(x,y\right), \end{array}$$

(4) $$\begin{array}{c} E_{\text{edge}}=1{\left|\nabla A\left(x,y\right)\right|}^{2}, \end{array}$$

(5) $$\begin{array}{c} E_{\text{line}}=-{\left(G_{\sigma }*\nabla^{2}A\right)}^{2}, \end{array}$$

(6) $$\begin{array}{c} E_{\text{term}}=\frac{\partial \theta }{\partial n_{⊥}}==\frac{\partial^{2}C/\partial n_{⊥}^{2}}{\partial C/\partial n}=\frac{{CyyC}_{X}^{2}-2CxyCxCy+{CxxC}_{y}^{2}}{{\left(C_{X}^{2}+C_{y}^{2}\right)}^{3/2}}. \end{array}$$

In equations (3)–(6), *E*_line_, *E*_edge_, *E*_term_, ∇, and *σ* stood for the line energy, edge energy, termination energy, gradient operator, and standard difference. Besides, *G*_*σ*_(*x*, *y*) meant the two-dimensional Gaussian equation.

Therefore, the minimum energy function was transformed into functional extremum, which should meet the Euler equation, as shown in the following equation:

(7) $$\begin{array}{c} \alpha L^{\prime \prime }\left(s\right)-\beta L^{\prime \prime \prime \prime }\left(s\right)-\nabla E_{\mathrm{ext}}=0. \end{array}$$

Further solution could be obtained as follows.

(8) $$\begin{array}{c} L_{t}\left(s,t\right)=\alpha L^{\prime \prime }\left(s,t\right)-\beta L^{\prime \prime \prime \prime }\left(s,t\right)-\nabla E_{\mathrm{ext}}, \end{array}$$

(9) $$\begin{array}{c} F_{\mathrm{int}}\left(L\right)+F_{\mathrm{ext}}\left(L\right)=0. \end{array}$$

In equations (8) and (9), *t* expressed the time, *s* represented the position, *F*_int_(*L*) = *αL*′′(*s*, *t*) − *βL*′′′′(*s*, *t*), and *F*_ext_(*L*) = −∇*E*_ext_.

The convergence process of Snake is shown in Figure 1. Its initial contour should be close to the actual boundary; otherwise, the convergence was wrong. The scope of external forces of the traditional Snake model was near the boundary but the direction of the sag lacked the effect of forces, and the active contour was difficult to converge to the sag.

A GCF gradient vector flow model was proposed in order to solve the Snake initialization and difficult convergence to the sag boundary, and its expression was *F*_ext_ = *B*(*x*, *y*), so −∇*E*_ext_ in equation (8) could be replaced with *B* (*x*, *y*).

(10) $$\begin{array}{c} L_{t}\left(s,t\right)=\alpha L^{\prime \prime }\left(s,t\right)-\beta L^{\prime \prime \prime \prime }\left(s,t\right)+B. \end{array}$$

Due to the fast convergence of traditional GVF-Snake, the final segmentation result had bumps and was not smooth enough. Therefore, the prior knowledge was introduced to combine, so as to achieve accurate segmentation. A large number of researches had proved that the prior knowledge-guided segmentation was more robust and accurate than other segmentation methods. Thus, the following improvements were made on the basis of equation (10).

(11) $$\begin{array}{c} L_{t}\left(s,t\right)=\alpha L^{\prime \prime }\left(s,t\right)-\beta L^{\prime \prime \prime \prime }\left(s,t\right)+\frac{1}{L\left(s,t\right)-C}\left(k_{1}B+k_{2}N\right). \end{array}$$

In equation (11), *B* and *N* stood for the gradient and normal vectors, respectively; *k*_1_ and *k*_2_ were constant coefficients; *F*_ext_(*L*) = 1/*L*(*s*, *t*) − *C*(*k*_1_*B* + *k*_2_*N*); *C* meant the contour center; 1/*L*(*s*, *t*) − *C* represented the weight coefficient of external force.

### 2.5. Observation Indexes

Relevant puncture indexes and surgical complications were recorded and compared among the patients in the two groups. The related indexes of puncture included times of puncture, puncture time, puncture depth, first puncture success rate, and pain incidence. Besides, puncture time referred to the time from the time when the puncture needle touched the patient's skin to the time when the puncture needle was removed. The successful puncture time would be recorded if the actual times of puncture were more than one. Possible complications during and after the surgery included nerve injury, hematoma, skin bruising, low back pain, presence of nerve root irritation, subarachnoid lapse, and infection.

### 2.6. Statistical Analysis

The SPSS19.0 version statistical software was used for analysis, and the measurement data could be expressed as mean ± standard deviation (*x̅*±*s*). In addition, the unpaired *t*-test and 2-dimensional analysis of variance were used for pairwise comparison, and *χ*^2^ test was employed to compare and analyze the count data between groups. *P* < 0.05 meant that the results were statistically substantial.

## 3. Results

### 3.1. Segmentation Results of Cervical Spine Magnetic Resonance Imaging-Based Image Segmentation Algorithm

20 MRI images were selected randomly, and 5 vertebrae were chosen from each image. Cervical spine MRI-based ISA was used for segmentation processing, and Dice Coefficient index was applied to evaluate the segmentation results of different MRI algorithms, as shown in Figure 2. Dice Coefficient was abbreviated as Dice, and its calculation equation is as follows.

(12) $$\begin{array}{c} \text{Dice}=\frac{2\left|A\cap B\right|}{\left|A\right|+\left|B\right|}. \end{array}$$

In equation (12), *A* represented the standard manual segmentation result and *B* meant the segmentation results of GVF-Snake or cervical spine MRI-based ISA. Dice obtained by solution was the ratio of the accurate segmentation part. The method was a mainly pixel method to calculate Dice.

Figure 2 indicates that the segmentation accuracies of traditional GVF-Snake algorithm were 89.2%, 88.2%, 84.1%, 78.4%, and 93.2, respectively. What is more, the segmentation accuracies of cervical spine MRI-based ISA were 95.5%, 92.3%, 98.3%, 98.4%, and 99.3% in sequence. Compared with the traditional GVF-Snake algorithm, the D-value of the cervical spine MRI-based ISA proposed in this study was obviously the highest, indicating that this algorithm was very effective and had marked improvement and better segmentation effects.

Conventional GVF-Snake algorithm and cervical spine MRI-based ISA were employed to segment MRI images, and the results are shown in Figure 3. It showed that there were protuberances in the segmentation region, and the segmentation results were not very smooth in the segmentation image with traditional GVF-Snake algorithm. In addition, some parts crossed the correct boundary to reach the strong boundary of another vertebra. The cervical spine MRI-based ISA had smoother segmentation results and better overall segmentation effect in contrast to the traditional GVF-Snake algorithm.

### 3.2. Clinical Data

Table 1 reveals the comparison results of clinical data among the patients in the two groups. There were 22 males and 14 females in group A aged 32.78 ± 9.36 years, with body mass index (BMI) of 21.56 ± 1.53 kg m^−2^, height of 164.32 ± 5.98 cm, and weight of 56.93 ± 7.87 kg. On the other hand, patients of group B included 20 males and 16 females, with an average age of 33.55 ± 10.05 years, BMI of 21.92 ± 1.24 kg m^−2^, height of 163.87 ± 4.76 cm, and weight of 57.36 ± 8.36 kg. It was known that there were no statistically obvious differences in gender, age, BMI, height, and weight among the subjects of groups A and B (*P* < 0.05).

### 3.3. Comparison on the Times of Puncture, Puncture Time, and Puncture Depth

Figure 4 indicates the comparison results of puncture times among the patients of groups A and B. There were 24 patients of group A with 1 time of puncture, 8 patients with 2 times of puncture, and 4 patients with 3 times of puncture. Besides, 16 patients of group B were punctured once, 12 patients were punctured 2 times, and 8 patients were punctured 3 times. The number of patients with 1 time of puncture in group A was greatly higher than that of group B (*P* < 0.05). The number of patients with 2 times in group A was obviously lower than that of group B (*P* < 0.05). In addition, the number of patients with 3 times in group A reduced sharply in contrast to group B (*P* < 0.05). Therefore, the difference was statistically considerable (*P* < 0.05) compared with the times of puncture in patients of groups A and B.

The comparison results of puncture time among patients in the two groups are shown in Figure 5. The puncture time of patients in group A was 9.9 ± 8.2 minutes, and that of group B was 15.2 ± 8.9 minutes. The puncture time of patients in group A was dramatically less than that of group B, with statistically substantial difference (*P* < 0.05).

Figure 6 reveals the comparison results of puncture depth among subjects of the two groups. The puncture depth of patients in group A was 53 ± 20 mm, and that of group B was 54 ± 24 mm. There was no huge difference in puncture depth of patients in groups A and B (*P* > 0.05).

### 3.4. Comparison of First Puncture Success Rate and Pain Incidence

Figure 7 shows the comparison results of first puncture success rate among the patients of the two groups. The first puncture success rates of patients in groups A and B were 78% and 54%, respectively. The success rate of the first puncture in patients of group A was considerably higher than that of group B, indicating there was a statistically obvious difference (*P* < 0.05).

Figure 8 shows a comparison of the incidence of puncture site pain between the two groups of patients. The incidence of pain at the puncture site was 6% in group A and 10% in group B. Therefore, the incidence of pain at the puncture site in group A was significantly lower than that in group B (*P* < 0.05).

### 3.5. Comparison of Complication Rates

The comparison results of complications among patients in the two groups are shown in Table 2. There were no patients of group A with epidural hematoma, infection, or subarachnoid injection during the puncture surgery, 4 patients with back pain (11.11%), and 4 patients with nerve root stimulation accounting for 11.11%. In group B, there were also no patients with epidural hematoma, infection, or subarachnoid injection during the puncture surgery, 17 patients with back pain (47.22%), and 12 patients with nerve root stimulation occupying 33.33%. The number of patients with back pain and nerve root irritation in group A was sharply lower than that of group B (*P* < 0.05).

The comparison results of complication rates among patients in the two groups are shown in Figure 9. The complication rates of patients in groups A and B were 22.22% and 80.56%, respectively. In addition, the complication rates of patients in group A were steeply lower than that of group B, with a statistically huge difference (*P* < 0.05).

## 4. Discussion

Cervical epidural puncture is an effective way to diagnose and treat acute and chronic pain diseases [12]. Compared with other sites, the tissue layer thickness of cervical epidural puncture site is increased, and the segment is relatively high, so the risk and difficulty of puncture during the actual operation is relatively high [13]. Traditional epidural puncture techniques rely mainly on the experience of pain physicians for positioning and puncturing [14]. During the entire operation, information such as the needle entry direction is nonvisual, and doctors check whether the patient's epidural space has reached through a series of experiments such as catheter insertion test, negative pressure test, and bubble efflux [15]. GVF-Snake is widely used in medical image segmentation, but it is insufficient in noise smoothing and edge protection, which greatly reduces the effect of medical image segmentation [16]. Therefore, it is of great significance to introduce prior knowledge to facilitate the segmentation performance of target images.

In this work, based on the traditional GVF-Snake algorithm and the existing knowledge, an ISA based on cervical spine MRI was proposed and applied to MRI image segmentation. The results showed that the segmentation result was smoother, the segmentation effect was better, and the segmentation accuracy was better than the GVF-Snake algorithm. This is consistent with the findings of Miri et al. [17], showing that cervical spine MRI-based ISA can improve the segmentation accuracy of medical MRI images.

Puncture time, puncture times, and puncture depth all affect the puncture success rate of cervical epidural puncture. Generally speaking, the puncture depth is relatively safe within 36 mm, while 54 mm is the average dangerous depth. Therefore, in actual surgery, caution should be exercised when the puncture depth exceeds 54 mm. In this work, the cervical spine MRI image segmentation algorithm was used to guide the cervical epidural puncture. The results showed that the puncture time of group A was 9.9 ± 8.2 (min), and in group B was 15.2 ± 8.9 (min), so the puncture time of patients in group A was significantly shorter than that of group B (*P* < 0.05). In addition, the incidence of pain at the puncture site of patients in group A was 6%, while that in in group B was 10%. The incidence of pain at the puncture site in group A was significantly lower than that in group B (*P* < 0.05). The success rate of the first puncture in group A was 78%, and that in group B was 54%. The success rate of the first puncture in group A was significantly higher than that in group B (*P* < 0.05). There was no significant difference in puncture depth between the two groups, indicating that ISA guidance based on cervical spine MRI can reduce the number of punctures, shorten the puncture time, reduce unnecessary injuries to patients, and improve the success rate, which is superior to the traditional blind puncture experience. This is consistent with the findings of Wybranski et al. [18]. The complication rate of group A was 22.22%, and that of group B was 80.56%. The incidence of complications in group A was significantly lower than that in group B (*P* < 0.05). Cervical spine MRI-based ISA guidance can reduce the risk of complications compared with the traditional blind puncture experience. It is in line with the findings of Shim et al. [19] and Nath et al. [20].

## 5. Conclusion

In this work, cervical spine MRI image segmentation algorithm was used to guide cervical epidural catheterization and used in the treatment of chronic pain. It was found that compared with traditional blind puncture, cervical spine MRI image segmentation algorithm guidance had a better application effect in the treatment of chronic pain with cervical epidural puncture and cannulation and can be applied in clinical practice. However, there were still some deficiencies in this work. For example, the number of samples was limited, the long-term efficacy of patients after surgery had not been discussed, and the cost of MRI measurement was high. In the follow-up, it was necessary to increase the number of samples and further analyze the impact on the prognosis of patients with chronic pain.

## Figures and Tables

**Figure 1:** Snake model.

**Figure 2:** Comparison of segmentation accuracy of different vertebrae with different algorithms.

**Figure 3:** MRI image segmentation results. (a) represented the image of the traditional GVF-Snake algorithm; (b) represented the image of the ISA based on cervical spine MRI, and the red box was the segmented image part.

**Figure 4:** Comparison of the number of punctures between group A and group B. ^∗^Compared with group A, *P* < 0.05.

**Figure 5:** Comparison of puncture time between patients in group A and group B. ^∗^Compared with group A, *P* < 0.05.

**Figure 6:** Comparison of puncture depth of patients in group A and group B.

**Figure 7:** The comparison of the success rate of the first puncture between the two groups of patients. ^∗^Compared with group A, *P* < 0.05.

**Figure 8:** Comparison of the incidence of pain at the puncture site between the two groups of patients. ^∗^Compared with group A, *P* < 0.05.

**Figure 9:** Comparison of the incidence of complications between the two groups of patients. ^∗^Compared with group A, *P* < 0.05.

**Table 1:** Comparison of clinical data of patients.

	Group A (*n* = 36)	Group B (*n* = 36)	*P*
Gender (male/female)	22/14	20/16	0.076
Age (years old)	32.78 ± 9.36	33.55 ± 10.05	0.329
BMI (kg m^−2^)	21.56 ± 1.53	21.92 ± 1.24	0.106
Height (cm)	164.32 ± 5.98	163.87 ± 4.76	0.383
Weight (kg)	56.93 ± 7.87	57.36 ± 8.36	0.866

**Table 2:** Comparison of complications among patients in the two groups (*n* (%)).

	Group A (*n* = 36)	Group B (*n* = 36)	*P*
Epidural infection	0 (0)	0 (0)	-
Epidural hematoma	0 (0)	0 (0)	-
Subarachnoid injection	0 (0)	0 (0)	-
Back pain	4 (11.11)	17 (47.22)	<0.05
Nerve root irritation	4 (11.11)	12 (33.33)	<0.05

## Data Availability

The data used to support the findings of this study are available from the corresponding author upon request.
